# NaHS Protects against the Impairments Induced by Oxygen-Glucose Deprivation in Different Ages of Primary Hippocampal Neurons

This article has been retracted.

**DOI:** 10.3389/fncel.2017.00067

**Published:** 2017-03-07

**Authors:** Qian Yu, Binrong Wang, Tianzhi Zhao, Xiangnan Zhang, Lei Tao, Jinshan Shi, Xude Sun, Qian Ding

**Affiliations:** ^1^Department of Anesthesiology, Tangdu Hospital, Fourth Military Medical UniversityXi’an, China; ^2^Department of Neurosurgery, Tangdu Hospital, Fourth Military Medical UniversityXi’an, China; ^3^Division of Scientific Research, Tangdu Hospital, Fourth Military Medical UniversityXi’an, China; ^4^Department of Anesthesiology, Guizhou Provincial People’s HospitalGuiyang, China

**Keywords:** NaHS, ischemia-reperfusion, ROS, apoptosis, neuroprotective, primary hippocampal neurons

## Abstract

Brain ischemia leads to poor oxygen supply, and is one of the leading causes of brain damage and/or death. Neuroprotective agents are thus in great need for treatment purpose. Using both young and aged primary cultured hippocampal neurons as *in vitro* models, we investigated the effect of sodium hydrosulfide (NaHS), an exogenous donor of hydrogen sulfide, on oxygen-glucose deprivation (OGD) damaged neurons that mimick focal cerebral ischemia/reperfusion (I/R) induced brain injury. NaHS treatment (250 μM) protected both young and aged hippocampal neurons, as indicated by restoring number of primary dendrites by 43.9 and 68.7%, number of dendritic end tips by 59.8 and 101.1%, neurite length by 36.8 and 66.7%, and spine density by 38.0 and 58.5% in the OGD-damaged young and aged neurons, respectively. NaHS treatment inhibited growth-associated protein 43 downregulation, oxidative stress in both young and aged hippocampal neurons following OGD damage. Further studies revealed that NaHS treatment could restore ERK1/2 activation, which was inhibited by OGD-induced protein phosphatase 2 (PP2A) upregulation. Our results demonstrated that NaHS has potent protective effects against neuron injury induced by OGD in both young and aged hippocampal neurons.

## Introduction

Stroke is now one of the leading causes of senior adult disability and death worldwide (Martin et al., 2005). Stroke is commonly caused by either interrupted or reduced blood supply to the brain such as ischemia, thereby leaving brain cells in a oxygen-glucose deprivation (OGD) condition. Even a short term of OGD can cause irreversibe damages to brain cells, while subsequent reperfusion, restoring blood supply to the brain, may aggravate the damage even further (Lin et al., 2016). Ischemia/reperfusion (I/R) induced oxidative stress, caused by impaired metabolism in the brain cells, is believed to be the one of the major contributors to brain I/R injury (Zeiger et al., 2009; Ma et al., 2015).

Ischemic preconditioning (IPC) is one of the protection mechanisms against I/R injury in the brian (Inokuchi et al., 2009; Zeiger et al., 2009). During I/R, the hypoxia-inducible factor 1 (HIF-1) pathway is activated, which downregulates the oxidative metabolism of brain cells by lowering the entry of metabolites into tricarboxylic acid (TCA) cycle, decreasing mitochondrial biogenesis and promoting reactive oxygen species (ROS) removal (Baxter et al., 2014). In aged brain cells with impaired mitochondria functions, ROS production was greatly increased compared with young brain cells (Della-Morte et al., 2013). Furthermore, gene expression profiles from mouse stoke model showed that transcriptional activity, axonogenesis, and neurogenesis were reduced in the peri-infarct area of aged animals, suggesting that the aged brain could respond to I/R injury transcriptionally (Signorini et al., 2014). Thus, there is an urgent need to search for promising neuroprotective agents, that could better protect ischemic neurons in the brain. Ideally, these new agents should prevent irreversible brain injury with minimal side effects, especially in the aged population, because IPC is more detrimental in the aged brain (Choe et al., 2009).

Hydrogen sulfide (H_2_S) is traditionally considered as a toxic gas with offensive odor. Recent studies revealed that H_2_S may exhibit multiple biological functions as a novel neural regulatory factor and a potential gaseous neuroprotector in both *in vitro* and *in vivo* model systems (Katayama et al., 2014). Our previous study suggested that sodium hydrosulfide (NaHS), an exogenous donor of H_2_S, exhibited potent protective effects against the brain I/R injury through inhibiting oxidative stress and apoptosis both *in vitro* and *in vivo* (Yu et al., 2015). However, questions remain whether NaHS exerts differential effects against insults on young and aged neurons. In the current study, we investigated the neuroprotective effects of NaHS treatment, as well as potential underlying mechanisms, in young and aged rat hippocampal neuron primary culture.

## Methods and Materials

### Primary Cultures of Hippocampal Neurons

Sprague-Dawley rats were provided by the Animal Center of Fourth Military Medical University. The care and use of animals in this study followed the guidelines and protocol approved by the Institutional Animal Care and Use Committee (IACUC) of Fourth Military Medical University. Primary cultures of hippocampal neurons were prepared as previously described (Brewer, 1997). In brief, the hippocampi from young (1 month, weighting 70–90 g) or aged Sprague-Dawley rats (24 months, weighting 500–600 g) were isolated and washed with dissecting fluid (PBS) on ice, then cut into 0.5 mm slices. Slices were minced and trypsinized (95% air and 5% CO_2_ at 37°C for 15 min), then 10% fetal calf serum (FCS)-containing Dulbecco’s Modified Eagle’s medium (DMEM) was applied to inactivate trypsin. After gentle trituration with a glass pipette, primary hippocampal neurons were dessociated, then mixed with DMEM supplemented with 20% FCS, filtrated, and eventually seeded at 1 × 10^9^ cell density on poly-*L*-Lysine-coated glass coverslips in 35 mm Petri dishes. NaHS were supplied into the culture media during the entire duration of culturing to the final indicated concentrations before examinations. For the control group, no NaHS was added in the culture medium.

### Oxygen-Glucose Deprivation (OGD)

Briefly, the medium of primary cultures of hippocampal neurons were replaced with pre-warmed Earle’s balanced salt solution (EBSS) without glucose. The cultures were incubated under the condition of 95% N_2_ and 5% CO_2_ at 37°C for 2 h as OGD (Ma et al., 2015).

### 3-(4,5-Dimethyl-2-thiazolyl)-2,5-diphenyl-2-H-tetrazolium Bromide (MTT) Assay

Cells were cultured in 96-well plates with or without NaHS for 7 days, then MTT was added at a final concentration of 0.5 mg/ml for 4 h. After the incubation, the medium was then replaced with DMSO to measure the blue MTT-formazan. The optical density (OD) were measured with BioTek’s Gen5^TM^ Microplate Readers (BioTek, Winooski, VT, USA).

### Lactate Dehydrogenase (LDH) Release Assay

Lactate dehydrogenase assay was performed as discribed before (Zeiger et al., 2009). Briefly, 2 × 10^4^ cells per well were seeded into 96-well plates in 100 μL culture medium and incubated at 37°C under 5% CO_2_ overnight. Then the plates were exposed to OGD or normal conditions for another 2 h. Fifty microliter of culture medium from each well was collected and centrifuged at 2,000 rpm for 5 min. The concentration of LDH in the supernatant of each well was measured using a LDH detection assay kit (Sigma, St. Louis, MO, USA) according to the manufacturer’s instructions.

### Immunostaining

Cells were immunostained and checked under a confocal microscope at indicated time points. Briefly, cells were fixed with 4% paraformaldehyde for 25 min and washed two times with PBS for 8 min. After permeabilization (0.1% Triton X-100, 15 min) and blocking (5% bovine serum albumin, 20 min), cells were stained with antibody against MAP-2 (Abcam, Cambridge, MA, USA) at room temperature for 2 h, then washed and incubated with the secondary antibodies for 1 h. Cells were then imaged by a scanning confocal microscope (Carl Zeiss, Germany).

### Western Blotting

Western blotting was performed according to previous descriptions (Yu et al., 2015). In brief, cells or nuclear fractions were lysed in lysis buffer [10 mM 4-(2-hydroxyethyl)-1-piperazineethanesulfonic acid, pH 7.4, 2 mM EGTA, 0.5% NP-40, protease inhibitors]. Twenty microgram equivalent total proteins were separated in a sodium dodecyl sulphate-polyacrylamide gel electrophoresis (SDS-PAGE) gel, then transferred to nitrocellulose membranes. Membranes were incubated with the primary antibodies against growth-associated protein (GAP)-43, phosphoryed-ERK1/2, total ERK1/2, PKA, PP2A or GAPDH (as an intenal control), followed by the corresponding horseradish peroxidase (HRP)-conjugated secondary antibodies (KPL, USA). All primary antibodies were purchased from Sigma, St. Louis, MO, USA. Immunoreactive bands were visualized with a chemiluminescence kit (Pierce, WI, USA). Intensities of protein bands were quantified by densitometry (Image J).

### Oxidative Stress Determination

Oxidative stress was measured by the activities of superoxide dismutase (SOD) and levels of malondialdehyde (MDA), nitric oxide (NO), and hydrogen peroxide. SOD activities were measured by SOD and Glutathione Peroxidase Assay Kits (Cayman Chemical, UK) according to the manufacturer’s instructions. MDA levels were determined by thiobarbituric acid reactive substances (TBARS) assay according to previously published method (Yu et al., 2015). NO levels were measured as total nitrite using Griess reagent with sodium nitrite as standard by a spectrophotometric method with measuring the absorbance at 540 nm. Glutathione (GSH), a major antioxidant, was quantified by high-performance liquid chromatography separation and fluorometric detection of the GSH-orthophthaldehyde adduct. Oxidized glutathione (GSSG) levels were obtained from substraction of the reduced GSH from the GSH values. F2-isoprostanes were quantified using a stable isotope dilution method with detection by gas chromatography/mass spectrometry.

### Characterization of Dendritic and Spine Phenotypes

At 7 days *in vitro* (DIV) of culturing, dendritic phenotypes were measured under a microscope precisely by the number of primary dendrites per cell, the number of dendritic end tips, and the average neurite length after the cells were immunostained as described before (Jugloff et al., 2005; Brandt et al., 2007). Spines are defined as subtle structures of hippocampal neurons, which emerge as small protrusions from the dendritic shafts. To analyze the effects of NaHS on spine formation of the neurons, hippocampal neuron cells were transfected with the mCherry-actin plasmid purchased from Addgene (Cambridge, MA, USA) using Lipofectamine 3000 (Invitrogen, Carlsbad, CA, USA) and then subjected to different conditions and treatments. Spines were visualized as described previously (Brewer, 1997) and the density was counted and expressed as number of spines per 10 μm of dendrites (Blanco-Suarez et al., 2014).

### Statistics

All statistical analyses were performed with GraphPad Prism software (GraphPad Software, USA). Values were obtained from at least three independent experiments, and presented as mean ± SD. Data were analyzed by one or two way ANOVA analysis followed by a Tukey’s *post hoc* test, with *P*-values < 0.05 considered statistical significant. ^∗^*P* < 0.05 and ^∗∗^*P* < 0.01 versus the corresponding controls are indicated.

## Results

### NaHS Protected OGD-Induced Impairments in Primary Cultures of Hippocampal Neurons Derived from Young and Aged Rats in a Dose-Dependent Manner

We first performed the colorimetric MTT assay to assess cell metabolic activity, and found that NaHS protected primary cultures of hippocampal neurons from OGD-induced cell damage in a dose-dependent manner (**Figures 1A,B**). Particularly, 250 μM of NaHS provided the best protection among groups of different concentrations ranging from 0 to 250 μM, whereas 1,000 μM of NaHS started to show cytotoxicity and reduced cell viability (**Figures 1A,B**). In our following experiments, we utilized 250 μM of NaHS due to its best protective effects. Notably, hippocampal neurons derived from aged rats showed more severe impairments than their young counterparts (**Figures 1A,B**), suggesting hippocampal neurons derived from aged rats were more vulnerable. In addition to MTT assay, we also performed the LDH release assay, a widely used enzymatic assay to assess cytotoxicity, and the results were consistent with our MTT assay, indicating that NaHS was able to protect the hippocampal neurons from OGD-induced cell damage (**Figure 1C**). Of note, when the cells were not subjected to OGD insult, 250 μM NaHS treatment had no obvious effects on cell viability and LDH release (Supplementary Figures S1A,B).

**FIGURE 1:** **Sodium hydrosulfide (NaHS) protects oxygen-glucose deprivation (OGD)-induced impairments in young and aged primary cultures of hippocampal neurons dose-dependently. (A)** Representative images of the young and aged cultures under 2 h OGD treatment in the presence of different concentrations of NaHS (0, 10, 50, 250, and 1,000 μM) for 7 days. Scale bar = 30 μm. **(B)** Relative cell viability of the cultures to control (no OGD and NaHS treatment) under OGD treatment following different NaHS treatment, measured by MTT assay. **(C)** Relative lactate Dehydrogenase (LDH) release to control in the experimental groups. Data were presented by the mean ± SD. ^∗^*p* < 0.05 and ^∗∗^*p* < 0.01 versus control, ^#^*p* < 0.05 and ^##^*p* < 0.01 versus OGD group.

### NaHS Treatment Significantly Repaired OGD-Induced Deficits in Neurite Sprouting and Outgrowth in Both Young and Aged Hippocampal Neurons

Dendrites are the primary sites of integrating synaptic input, and dendritic branching plays an essential role in neuronal circuit formation. The neurite sprouting and outgrowth were examined in the cultured hippocampal neurons. OGD insult inhibited the sprouting and outgrowth at 7 DIV, while 250 μM NaHS treatment rescued these impairments (**Figure 2A**). The number of primary dendrites per cell (**Figure 2B**), dendritic end tips (**Figure 2C**), and the average neurite length (**Figure 2D**) were also reduced following OGD insult, while 250 μM NaHS rescued the above OGD-induced impairments, supporting the protective role of NaHS treatment. Similarly, 250 μM NaHS treatment did not affect neurite sprouting and growth when the cells were not subjected to OGD insult (Supplementary Figures S1C–E).

**FIGURE 2:** **Sodium hydrosulfide treatment (250 μM) could significantly repair OGD-induced injuries of neurite sprouting and outgrowth in the young and aged hippocampal neurons in 7 DIV. (A)** Typical hippocampal neurons with extending neurites in the cultures, stained for MAP-2. Scale bar = 40 μm. The neurite sprouting and outgrowth were analyzed by the number of primary dendrites per cell **(B)**, the number of dendritic end tips **(C)**, and the average neurite length **(D)**. Data were presented by the mean ± SD. ^∗^*p* < 0.05 and ^∗∗^*p* < 0.01 versus corresponding control, ^##^*p* < 0.01 versus corresponding OGD group.

### NaHS Treatment Partially Restored the OGD-Induced Loss of Spine Density in Both Young and Aged Hippocampal Neurons

Following dendritic tree elaboration, morphologically specialized spines emerge as small protrusions from the dendritic shafts, which represent the main postsynaptic compartment to receive excitatory inputs. As shown in **Figure 3A**, spine density was impaired by OGD insults in both young and aged hippocampal neurons at 14 DIV. Further NaHS treatment (250 μM) partially rescued the OGD-induced spine density reduction (**Figure 3A**). By quantifying the spine density as number of spines per 10 μm of dendrites, we further confirmed that OGD insults significantly reduced the spine density, which could be restored by NaHS treatment (**Figure 3B**).

**FIGURE 3:** **Sodium hydrosulfide treatment (250 μM) partially restores the loss of spine density induced by OGD insult in both young and aged hippocampal neurons in 14 DIV. (A)** The cultures were transfected with mCherry-actin and observed. Scale bar = 2 μm. The spines could be clearly seen in the experimental groups. **(B)** Spine density was expressed as number of spines per 10 μm of dendrites. Data were presented by mean ± SD. ^∗^*p* < 0.05 and ^∗∗^*p* < 0.01 versus corresponding control (no treatment), ^##^*p* < 0.01 versus corresponding OGD group.

### NaHS Treatment Inhibited the OGD-Induced GAP-43 Downregulation in Both Young and Aged Hippocampal Neurons

Growth-associated protein-43 is a membrane-bound protein that functions to promote neurite regeneration and outgrowth after nerve injury (Frey et al., 2000). Effects of NaHS on GAP-43 expressions in young and aged hippocampal neurons were examined at 3 and 7 DIV (**Figure 4A**). Levels of GAP-43 were reduced by OGD insults in both young and aged hippocampal neurons, and NaHS treatment (250 μM) could reverse the downregulated GAP-43 expressions (**Figure 4B**), suggesting that NaHS may acted through the downstream effector GAP-43 to restore the OGD-impaired neurite growth. In addition, effect of NaHS on GAP-43 expression was also significantly more profound at 7 DIV.

**FIGURE 4:** **Effects of NaHS (250 μM) on growth-associated protein (GAP)-43 expressions in young and aged hippocampal neurons in 3 or 7 DIV. (A)** Western blot analysis of GAP-43 (MW: 43 kDa) under OGD insult and NaHS treatment. GAPDH (MW: 37 kDa) was used as a loading control. **(B)** Relative GAP-43 expressions in the experimental groups when compared to control. Data were presented by mean ± SD. ^∗^*p* < 0.05 and ^∗∗^*p* < 0.01 versus corresponding control (no treatment), ^##^*p* < 0.01 versus corresponding OGD group.

### NaHS Treatment Attenuated OGD-induced Oxidative Stress in both Young and Aged Hippocampal Neurons

During cerebral I/R, abundant free radicals are produced to provoke oxidative stress, which contributes to neuronal apoptosis and ischemic brain damage after stroke (Chen et al., 2011). The importance of oxidative stress prompted us to examine the relative SOD activity, MDA levels, NO levels, and hydrogen peroxide levels. SOD is an antioxidant enzyme mediating defense against oxidative stress. MDA is a marker for oxidative stress, while NO and hydrogen peroxide are ROS released under oxidative stress (Evereklioglu et al., 2003). Our results demonstrated that the relative SOD activity and GSH levels were reduced by OGD insults, which can be rescued by NaHS treatment, in both young and aged hippocampal neurons (**Figures 5A,E**). While on the other hand, the levels of MDA, NO, hydrogen peroxide, GSSG, and F_2_-isoprostanes were elevated by OGD insults, and subsequently inhibited by NaHS treatment (**Figures 5B,C,D,F,G**, respectively). Taken together, OGD-induced severe oxidative stress, which could be attenuated by NaHS treatment in both young and aged hippocampal neurons. Interestingly, NaHS treatment (250 μM) attenuated OGD-induced increase in protein carbonyls contents in both young and aged hippocampal neurons 3 h after re-oxygenation (**Figure 5H**).

**FIGURE 5:** **Sodium hydrosulfide (250 μM) successfully attenuates OGD-induced oxidative stress in both young and aged hippocampal neurons.** Oxidative stress was characterized by determining the relative superoxide dismutase (SOD) activity **(A)**, malondialdehyde (MDA) levels **(B)**, nitric oxide (NO) levels **(C)**, hydrogen peroxide levels **(D)**, glutathione (GSH) levels **(E)**, oxidized glutathione (GSSG) levels **(F)**, and F_2_-isoprostanes **(G)** to control. **(H)** NaHS treatment (250 μM) also attenuates OGD-induced increase of protein carbonyls contents in both young and aged hippocampal neurons 3 h after re-oxygenation. Data were presented by mean ± SD. ^∗^*p* < 0.05 and ^∗∗^*p* < 0.01 versus corresponding control (no treatment), ^#^*p* < 0.05 and ^##^*p* < 0.01 versus corresponding OGD group.

### ERK Signaling Was Involved in the Neuroprotection of NaHS

Since NaHS acted as antioxidant, we further studied its association with the ERK pathway, which was reported to have a neuroprotective role against oxidative stress (Gu et al., 2009). Dynamic interplay between kinases and phosphatases is critical for the regulation of ERK signaling, and ERK1/2 is known to be activated by phosphorylation. Our Western blot revealed that OGD treatment inhibited expressions of phosphorylated-ERK1/2 in both young and aged hippocampal neurons, while subsequent 250 μM NaHS treatment could restore ERK1/2 phosphorylation, as quantified using GAPDH (**Figures 6A,B**). The quantification results using total ERK1/2 as normalization was consistent with that using GAPDH (data not shown). PP2A and PKA are the two major enzymes responsible for ERK1/2 phosphorylation. The levels of PKA were not affected by either OGD or NaHS treatment (**Figures 6C,D**). However, PP2A levels were upregulated by OGD treatment, which were then restored to control levels by NaHS (**Figures 6E,F**), indicating OGD-induced PP2A to dephosphorylate ERK1/2 and inhibit ERK signaling, while NaHS treatment restored PP2A expression to control levels.

**FIGURE 6:** **Involvement of ERK pathway in the neuroprotection of NaHS. (A,B)** OGD treatment inhibited p-ERK1/2 (MW: p-ERK1/2, 44/42 kDa; EKR1/2, 44/42 kDa) expression in both young and aged hippocampal neurons, while 250 μM NaHS could increase ERK1/2 phosphorylation, characterized by western blot analysis. **(C,D)** Western blotting shows that there was no significant difference in PKA (MW: 45 kDa) levels between the experimental groups. **(E,F)** OGD increased PP2A (MW: 35 kDa) expressions, while NaHS decreased its expressions. The expression levels from each group were normalized to those of GAPDH (as a loading control, MW: 37 kDa) and are presented as ratios to control. Data were presented by mean ± SD. ^∗^*p* < 0.05 and ^∗∗^*p* < 0.01 versus corresponding control (no treatment), ^##^*p* < 0.01 versus corresponding OGD group.

## Discussion

During the process of aging, toxins generated by the sustaining metabolism accumulate in long-living cells such as neurons (Calabrese et al., 2012). The accumulated toxic metabolic products could inhibit mitochondrial ATP turnover in neuron cells, leading to “aged” mitochondria with impaired ATP production and increased ROS leakage (Martin et al., 2005). ROS is a well known factor contributing to brain I/R injury (Zeiger et al., 2009; Ma et al., 2015). During I/R, the brain activates its own protection mechanism IPC to remove the ROS generated by I/R injury. Whereas in aged brain cells with “aged” mitochondria, IPC function is significantly impaired, making the aged brain cells more vulnerable to I/R injury. Thus, the search for promising neuroprotective agents for stoke treatment in elder patients has attracted increasing research attention.

There has been a line of studies documenting the neuroprotective effects of H_2_S. For instance, H_2_S could slow down progression of Alzheimer’s disease in various animal models (Giuliani et al., 2013), as well as attenuate hypoxia-induced neurotoxicity through inhibiting microglial activation (Zhang et al., 2014). In addition, prolonged exposure to H_2_S was able protect the aged rat brain from cerebral injury, by inhibiting the upregulation of phagocytosis-specific protein annexin 1 (Joseph et al., 2012). Similarly, Sandu and colleagues have recently reported that post-stoke H_2_S treatment increased vascular density, reduced brain infarction and inflammation in aged ischemic rat model (Sandu et al., 2016a,b). As expected, being a donor of H_2_S, NaHS was also widely reported to exhibit beneficial physiological effects in the brain. As early as 1990, Warenycia and colleagues first discovered that chronic NaHS treatment could prevent the stress-induced increases in amino acid levels in brainstem of rats (Warenycia et al., 1990). Furthermore, exogenous NaHS could affect the cAMP signaling pathway and attenuate naloxone-precipitated withdrawal syndromes in the nucleus accumbens of heroin-dependent rats (Jiang et al., 2012). NaHS was also reported to prevent hypoxia-induced behavioral impairment in neonatal mice (Wang et al., 2013). Using a rat model of cardiac arrest and cardiopulmonary resuscitation (CPR), Pan et al. (2014) found that administration of NaHS ameliorated neurological dysfunction likely by preserving and promoting mitochondrial biogenesis in the brain. Two recent studies, including our own, have also shed light on the molecular mechanism underlying the beneficial effects of NaHS, which involves both the PARP/AIF and MAPK/NF-κB pathways (Liu et al., 2015; Yu et al., 2015).

In the current study, we investigated the effects of NaHS against I/R injury in young and aged rat primary hippocampal neurons. We first developed primary cultures of hippocampal neurons from differentially aged rats, and then investigeated the effects of NaHS on the primary neurons under OGD condition. Aged neurons showed more severe OGD-induced impairments, compared with their young counterparts (**Figure 1**), which is consistent with the clinical observation that elder patients have worse outcome during I/R injury. NaHS exhibited dose-dependent protective effects on both young and aged neurons during OGD stress. Two hundred fifty micrometer NaHS provided the best protection among concentrations ranging from 0 to 250 μM, whereas 1,000 μM NaHS started to show cytotoxicity and reduced cell viability (**Figures 1A,B**), suggesting appropriate dose application of NaHS should be taken into consideration for future treatment. I/R injury induced cell death is mostly due to cell necrosis leading to cellular organelle swelling, plasma membrane disruption, and release of intracellular contents (Choe et al., 2009). Therefore, the extent of cell necrosis can be quantified by measuring the release of the intracellular enzyme LDH (Zeiger et al., 2009). We then performed LDH releasing assay to examine the effects of NaHS on neuron cell necrosis during OGD. Indeed, NaHS could significantly inhibit LDH releasing from both young and aged neurons in a dose-dependent manner, suggesting NaHS inhibited the neuron cell necrosis following OGD.

Dendrites are the primary sites of integrating synaptic inputs, and neurite sprouting and outgrowth play critical roles in neuronal circuit formation. Morphologically specialized spines are subtle structures dendrites, which appear as small protrusions from the dendritic shafts, and are important for excitatory inputs. Upon close observation, we discovered that the complex morphology of hippocampal neurons was impaired by OGD-induced injuries at 7 DIV, in terms of reduced numbers of primary dendrites per cell, fewer dendritic end tips, shorter average neurite, and lower spine density (**Figure 2, 3**). The findings are consistent with previous reports that OGD inhibited neurite outgrowth (Orban-Gyapai et al., 2014) and induced spine shrinkage (Blanco-Suarez et al., 2014). NaHS treatment successfully rescued the normal morphology of OGD-treated neurons, indicating proper synaptic input was restored. GAP-43 is a membrane-bound protein that can promote the regeneration and outgrowth of neurite after nerve injury (Frey et al., 2000). NaHS treatment could promote GAP-43 after OGD insults, suggesting GAP-43 might be a downstream effector of NaHS treatment.

Since NaHS is an exogenous donor of H_2_S, which regulates oxidant balance, we speculated that NaHS might regulate the oxidant balance in neuron cells after OGD insults. We measured the levels of MDA, NO and hydrogen peroxide and the relative SOD activity in neuron cells under OGD condition with or without NaHS treatment. Indeed, the relative SOD activity was reduced by OGD insults, which could be rescued by NaHS treatment in both young and aged neurons. Furthermore, the levels of MDA, NO, and hydrogen peroxide were significantly elevated by OGD insults, and subsequently inhibited by NaHS treatment as well. Recent studies have shown that ROS have multiple biological functions other than directly damaging brain cells during I/R injury, such as activating the HIF-1 pathway which is critical to the IPC (Wang et al., 2015; Lin et al., 2016). In aged brain cells, these ROS-induced protective signaling pathway can be activated transcriptionally, but are eventually inhibited (Signorini et al., 2014). Moreover, recent studies also suggested that lower concentrations of H_2_S exhibited antioxidant effects, whereas higher concentrations may cause genotoxicity (Katayama et al., 2014), consistent with the protective effect of low dosage NaHS against I/R damage and cytotoxicity of higher concentration.

ERK pathway has been reported to exhibit neuroprotective effects against oxidative stress in brain cells of patients with Parkinson’s disease (PD) (Gu et al., 2009). ERK1/2 signaling is regulated through a dynamic interplay between kinases and phosphatases. The activation of ERK signaling pathway, as a result of ERK1/2 phosphorylation, is critical for protecting brain cells against oxidative stress in PD and/or I/R injury. In the current study, expressions of phosphorylated-ERK1/2 in neurons were downregulated by OGD, which could then be rescued by NaHS treatment, suggesting the involvement of ERK pathway in the neuron protective effects of NaHS as well.

Many other studies demonstrated the protective effects of NaHS during oxidative stress in different organs. For example, Dong et al. (2015) used NaHS to inhibite the mitochondrial apoptosis pathway, and successfully prevented cochlear hair cells from gentamicin-induced cell death (Dong et al., 2015). Of particular interest to our current research, the administration of NaHS demonstrated promising effects in significantly ameliorating I/R injury in multiple organs including the brain (Kimura et al., 2010; Yin et al., 2013), the heart (Johansen et al., 2006; Lin et al., 2016), the intestines (Liu et al., 2009, 2012), the kidney (Azizi et al., 2015; Ibrahim et al., 2015), and the liver (Kang et al., 2009; Tu et al., 2016). OGD increases oxidative stress, while NaHS presents as a promising antioxidant to attenuate oxidative stress, especially in aged neurons. Our current study adds NaHS, an exogenous donor of H_2_S, into the list of antioxidant agents that could potentially treat aged neurons against I/R induced injuries.

In summary, we hereby report that NaHS treatment exerts neuroprotective effects on both young and aged hippocampal neurons in a dose-dependent manner, preventing them from OGD-induced impairments. OGD insults damage the neurite sprouting and outgrowth, while NaHS treatment can alleviate damages to the neurons by restoring number of primary dendrites by 43.9 and 68.7%, number of dendritic end tips by 59.8 and 101.1%, neurite length by 36.8 and 66.7%, and spine density by 38.0 and 58.5% in the OGD-damaged young and aged neurons, respectively. Notably, even though aged neurons are more vulnerable than young neurons, NaHS treatment still provides apparent protection for aged neurons. Furthermore, neuroprotective effects of NaHS treatment is likely to involve the oxidative stress and the ERK pathway.

## Author Contributions

Conceived and designed experiments: QD. Provided reagents: XS. Performed experiments: QY, BW, TZ, XZ, LT, and JS. Analyzed the data: QY and BW. Wrote the paper: XS and QD.

## Conflict of Interest Statement

The authors declare that the research was conducted in the absence of any commercial or financial relationships that could be construed as a potential conflict of interest.
